# Application of Machine Learning in Rheumatic Immune Diseases

This article has been retracted.

**DOI:** 10.1155/2022/9273641

**Published:** 2022-01-25

**Authors:** Yuan Li, Linru Zhao

**Affiliations:** Department of Rheumatology, Tianjin First Central Hospital, Tianjin 300192, China

## Abstract

People are paying greater attention to their personal health as society develops and progresses, and rheumatic immunological disorders have become a serious concern that affects human health. As a result, research on a stable, trustworthy, and effective auxiliary diagnostic method for rheumatic immune disorders is critical. Machine learning overcomes the inefficiencies and volatility of human data processing, ushering in a revolution in artificial intelligence research. With the use of big data, machine learning-based application research on rheumatic immunological disorders has already demonstrated detection abilities that are on par with or better than those of medical professionals. Artificial intelligence systems are now being applied in the field of rheumatic immune disorders, with an emphasis on the identification of patient joint images. This article focuses on the use of machine learning algorithms in the diagnosis of rheumatic illnesses, as well as the practical implications of disease-assisted diagnosis systems and intelligent medical diagnosis. This article focuses on three common machine learning algorithms for research and debate: logistic regression, support vector machines, and adaptive boosting techniques. The three algorithms are used to build diagnostic models based on rheumatic illness data, and the performance of each model is assessed. According to a thorough analysis of the assessment data, the diagnostic model based on the limit gradient boosting method has the best resilience. This article presents machine learning's use and advancement in rheumatic immunological disorders, as well as new ideas for investigating more appropriate and efficient diagnostic and treatment techniques.

## 1. Introduction

According to the World Health Organization, more than 3 million Chinese people die prematurely every year, dying from various noncommunicable diseases before the age of 70. Furthermore, more than 70% of white-collar workers in mainland China's cities are in poor health, with more than 60% being overworked, and their health is visibly poor. Rheumatic immune disorders continue to be common among them. As a result, one of the most important factors in improving people's quality of life, protecting their health, and increasing their life expectancy is the creation of medical standards. The following are the current major issues in China's medical business [1, 2]: Medical resources are extremely limited, and inhabitants have a difficult time seeing a doctor. China currently has 20% of the world's population but only 2% of global medical resources. Furthermore, medical resources in the United States are distributed inequitably. Many high-quality resources are concentrated mostly in large cities and coastal locations, yet large formal hospitals are difficult to come by in many economically poor places. The difficulty of seeing a doctor is strongly related to the paucity of medical resources, particularly of extremely high-quality medical resources [3]. For a long time, the lack of a uniform doctor education and training system, as well as professional evaluation criteria, has resulted in a lack of consistency in medical standards and the inability to effectively diagnose patients' conditions. Furthermore, the doctor-to-patient ratio is significantly skewed. Overworked clinicians are more likely to make mistakes that prolong the patient's recovery [4]. As a result, another significant issue confronting our country's medical business is the speedy and precise diagnosis of diseases. Medical informatization is lacking, and diagnosing technology is outdated. Internationally, medical informatization is a prominent development trend. In recent years, as the medical system's reform has progressed, the informatization infrastructure has reached an advanced stage of development.

China's medical informatization level is still at the essential information management system and registration fee system, disease diagnosis is still primarily manual, diagnostic accuracy cannot be guaranteed, and efficiency is low. Another critical success in changing the status quo of our country's medical business has been speeding up the development of medical informatization and boosting the quality and efficiency of medical services [5, 6]. The aforementioned issues have hampered the development of the medical business while also affecting domestic social stability and people's living conditions.

Machine learning (ML) is an interdisciplinary subject based on computer science and mathematics that integrates cybernetics, information theory, determinism, and other theories, methods, technologies, and application systems to simulate, extend, and expand human intelligence theories, technologies, and application systems. In recent years, China has been a big supporter of artificial intelligence development and application in medical imaging-assisted diagnostics. The rate of auxiliary diagnosis of bone, lung, cardiovascular, and cerebrovascular illnesses has grown thanks to the standardization of medical imaging data gathering. In 2019, Nature Medicine published eight papers focusing on the use of artificial intelligence in medicine, including the early detection of diseases such as diabetic retinopathy, the diagnosis of benign and malignant skin lesions, the determination of histopathological types of lung cancer, and the diagnosis of radius and hip fractures. However, there are currently few research efforts on artificial intelligence in rheumatic immunological illnesses, with most of them focused on diseases like SLE and being single-center small-sample studies. One of the future research directions is to use artificial intelligence technology to improve the diagnosis rate and prognosis of rheumatic immunological disorders. Furthermore, because rheumatic immune illnesses can impact various organs, artificial intelligence research in other diseases can be applied to develop an artificial intelligence research system for rheumatism.

One of the hottest research directions is the AI-based disease-assisted diagnosis system [7]. There have been numerous studies of machines being used to diagnose patients both at home and abroad in recent years, and they have worked admirably [8–11]. The disease-assisted diagnostics method outperforms the competition in addressing issues, such as the lack of medical resources and outdated diagnostics. Machine learning aims to improve a machine's performance by drawing on previous experience and data. It can actively learn from sample data and make high-accuracy decisions as a result. Hence, it has been extensively investigated and used in disease diagnosis. In this article, we focus on applying machine learning algorithms in the diagnosis of rheumatic immune diseases.

## 2. Related Work

Ledley et al. [12] were among the first to introduce mathematical, statistical models into clinical medicine, and they advocated employing mathematical-statistical models as a tool for computer-aided diagnosis systems in the late 1950s. Medical expert systems have been the dominant tool for disease diagnosis since the 1960s. MYCIN [13], for instance, is a medical expert system for identifying and treating infectious diseases. Fu and Chen [14] introduced CADIAG, a rule-based fuzzy expert system to identify rheumatic and pancreatic disorders. Chiarugi et al. [15] proposed a heart failure decision support system that uses Bayesian and other statistical approaches to identify diseases and is based on a fuzzy logic disease diagnosis system. These medical expert systems primarily perform medical diagnoses based on clinical knowledge and diagnosis experience from medical experts. The process of disease diagnosis, on the other hand, will grow complicated and unstable due to the diversity and instability of diseases. Traditional medical expert systems are mechanized to gather information and experience from medical experts, who are inherently subjective. In diagnostic applications, there are several limits.

Machine learning theory and technological advancements offer a promising direction for disease-assisted diagnosis systems. Many disease-assisted diagnosis systems based on machine learning classifiers have arisen to assist medical staff in diagnosing and evaluating diseases, improving medical quality, reducing medical costs, and controlling diagnosis costs. For example, Yuan et al. [16] developed a support vector machine (SVM) classifier to aid in the diagnosis of cancer using the content of macro and trace components in human blood in 2007. Multiple classifiers were combined in the auxiliary detection of tuberculosis by Han et al. [17] in 2012.

Machine learning is a branch of artificial intelligence that can be separated into three stages of growth [18–23].

1. Budding period: from the mid-1950s to the mid-1960s, people attempted to pass programming to control the computer to obtain logical reasoning ability and then make the machine have specific thinking abilities. The machine's inference results, on the other hand, fell significantly short of people's expectations. Many studies have discovered that having artificial intelligence with logical reasoning capabilities is insufficient and that a considerable quantity of prior knowledge is required.
2. Development period: during the development period, individuals attempted to guide computers to make judgments and conclusions based on artificial rules from the mid-1960s to the mid-1980s. Expert systems came in a variety of forms, but they all suffered from the problem of limited knowledge. In other words, individuals were unable to find universal laws that would allow them to address the seemingly infinite problem of knowledge and information. As a result, researchers began to investigate how to teach robots to learn on their own.
3. Prosperous period: machine learning has ushered in accelerated development with the rise of the Internet and technology from the 1980s to the present, throughout the affluent period, and many learning algorithms have continued to emerge. Simultaneously, the rapid advancement of machine learning has aided the establishment of new areas, such as pattern recognition and data mining.

Since its inception, machine learning has been split into supervised learning, unsupervised learning, and semisupervised learning. The input parameters and output results of the specified training data are necessary in supervised learning. The output result has been arbitrarily demarcated in advance among them. Supervised learning is mostly focused on classification and regression methods to develop predictive models that can forecast continuous and discrete data. Linear regression, support vector machines, logistic regression, decision trees, random forests, K-nearest neighbors, boosting algorithms, and artificial neural networks are all examples of supervised learning techniques.

The primary distinction between unsupervised and supervised learning is that no output results are required in the training set in unsupervised learning. Clustering and dimensionality reduction are two standard unsupervised learning techniques, and their primary goal is to discover regularity in the training data.

Semisupervised learning combines supervised and unsupervised learning methods. It classifies unlabeled data using labeled data. This is the method to utilize when only a small number of output results need to be identified. Machine learning is now widely employed in various industries, including medicine, media, and automobiles, because of its rapid progress in recent decades. Machine learning has spawned many subdisciplines, including data mining, deep learning, pattern recognition, remote sensing, and information security.

## 3. Methods

Machine learning is a multifield interdisciplinary study that encompasses various topics, including probability theory, statistics, and approximation theory. Its core concept is to utilize mathematical reasoning and machine learning algorithms to let machines extract meaningful rules from data and use those rules to predict unknown data. The classification of disease diagnosis using machine learning, which is part of the classification prediction of supervised learning, is the subject of this paper's research. The three machine learning classification algorithms discussed in the article will be explained in detail in this section.

### 3.1. Logistic Regression

The logistic regression model is mostly used to solve problems involving binary classification detection. In epidemiology, logistic regression models are increasingly being used to forecast the likelihood of developing a disease based on the disease's risk factors.

Assuming that the random variable *X* obeys the logistic distribution, the cumulative distribution function (CDF) of *X* is as follows:

(1) $$\begin{array}{c} F\left(x\right)=\frac{1}{1+\text{exp}\left(-\left(x-\mu \right)/\gamma \right)}. \end{array}$$

The probability density function (PDF) of *X* is as follows:

(2) $$\begin{array}{c} f\left(x\right)=\frac{\text{exp}\left(-\left(x-\mu \right)/\gamma \right)}{\gamma {\left(1+\exp\left(-x-\mu /\gamma \right)\right)}^{2}}, \end{array}$$

where *μ* is the position parameter and *γ* is the shape parameter.

The cumulative function of the logistic distribution is an S-shaped curve, so the logistic distribution is also called the Sigmoid distribution. The function curve is symmetric about the center of the point (*μ*, 0.5); that is, it satisfies

(3) $$\begin{array}{c} F\left(\mu -x\right)+\left(\mu +x\right)=1. \end{array}$$

In this article, disease diagnosis and prediction constitute a binary classification problem, so the article will mainly introduce the binomial logistic regression model. A conditional probability distribution represents the binomial logistic regression model. The independent variable is the input variable whose value is the m-dimensional real vector space *R*^*m*^, and the dependent variable is the output variable *Y* whose values are 1 and 0. The conditional probability distribution of the model is as follows:

(4) $$\begin{array}{c} P\left(Y=1\;|X=x\right)=\frac{\text{exp}\left(wx+b\right)}{1+\text{exp}\left(wx+b\right)},\\ P\left(Y=0\;|X=x\right)=\frac{1}{1+\text{exp}\left(wx+b\right)}, \end{array}$$

where *w* is weight vector. The weight vector parameter and the bias parameter are placed together and still recorded as *w*. At this point, the binomial logistic regression model can be written as

(5) $$\begin{array}{c} P\left(Y=1\;|X=x\right)=\frac{\text{exp}\left(wx\right)}{1+\text{exp}\left(wx\right)},\\ P\left(Y=0\;|X=x\right)=\frac{1}{1+\text{exp}\left(wx\right)}. \end{array}$$

When the input variable is given and the parameter is known, the probability that the output parameter is 1 and 0 can be obtained through the formula. Then, we judge the output parameter *Y* according to the preset threshold *v*. Normally, the threshold value is *v*=0.5.

Generally, maximum likelihood estimation is used to solve the to-be-estimated parameters of the Logit regression model. Here, suppose

(6) $$\begin{array}{c} P\left(Y=1\;|X=x\right)=\pi \left(x\right),\\ P\left(Y=0\;|X=x\right)=1-\pi \left(x\right). \end{array}$$

For the training data set of *n* sample points, the likelihood function is

(7) $$\begin{array}{c} L\left(w\right)=\overset{n}{\underset{i=1}{\prod }}{\left[\pi \left(x_{i}\right)\right]}^{y_{i}}{\left[1-\pi \left(x_{i}\right)\right]}^{1-y_{i}}. \end{array}$$

Therefore, the log likelihood function is

(8) $$\begin{array}{c} l\left(w\right)=\text{ln}\left(L\left(w\right)\right). \end{array}$$

Then, by solving the maximum value of *l*(*w*), the estimated parameter $\hat{w}$ can be obtained. When solving $\hat{w}$, the gradient iteration method or Newton iteration method is generally used. At this time, the estimated binomial Logit regression model is

(9) $$\begin{array}{c} P\left(Y=1\;|x\right)=\frac{\text{exp}\left(\hat{w}x\right)}{1+\text{exp}\left(\hat{w}x\right)},\\ P\left(Y=0\;|x\right)=\frac{1}{1+\text{exp}\left(\hat{w}x\right)}. \end{array}$$

For a given instance, the output parameter *Y* of the instance can be predicted according to the above formula.

### 3.2. Support Vector Machine

The support vector machine (SVM) concept was developed in the 1960s. The support vector machine is a two-class classification model that addresses tiny samples, nonlinear patterns, and high-dimensional pattern recognition. It has become one of the hottest study subjects in the present machine learning field, with applications in various fields. The theoretical basis of SVM is the Vapnik–Chervonenkis (VC) dimension and structural risk minimization (SRM) principles in statistical learning theory [24–26]. The VC dimension is a fundamental concept in machine learning, which provides a solid theoretical foundation for the learnability of many machine learning methods. The relevant definition of the VC dimension is as follows: For an indicator function set, there are at most sample points that can be broken up in all possible forms by the OPERATION of the function set, then is the VC dimension of the function set. If the number of samples H can take any value, the VC dimension of the function set is infinite. The VC dimension is a judgment on the learning ability and complexity of the model. The larger the VC dimension, the stronger the model learning ability and the higher its complexity.

The structural risk minimization strategy is to control the expected risk of the model in the sample. In other words, the role of SRM is to prevent the model from overfitting. Before discussing SRM, we must first introduce the principle of empirical risk minimization (ERM).

For a given training data set, where each sample point is composed of an instance *X* and a label *Y*, the empirical risk of the model is expressed as

(10) $$\begin{array}{c} R_{emp}\left(f\right)=\frac{1}{n}\overset{n}{\underset{i=1}{\sum }}l\left(y_{i},f\left(x_{i},\omega \right)\right), \end{array}$$

where *ω* is generalized parameters of the model and *l* is the loss function.

Under the principle of empirical risk minimization, we can consider that the average loss of the optimal model has reached the minimum, which is

(11) $$\begin{array}{c} f=\arg\min\;R_{emp}\left(f\right). \end{array}$$

The notion of empirical risk minimization can have a good learning impact for large sample data. The notion of empirical risk minimization, on the other hand, frequently leads to overfitting for small-sample data. It is advised that structural risks be minimized to avoid this occurrence. The definition of structural risk is as follows:

(12) $$\begin{array}{c} \;R_{arm}\left(f\right)=\;R_{emp}\left(f\right)+\lambda J\left(f\right), \end{array}$$

where *λ* is penalty factor and *J*(*f*) is the complexity of the model.

Structural risk is equal to empirical risk plus confidence risk. Generally, under the SRM principle, we can consider that the structural risk of the optimal model has reached a minimum, which is

(13) $$\begin{array}{c} f=\arg\min\;R_{srm}\left(\omega \right). \end{array}$$

Models with low structural risk tend to have good prediction effects on both the training set and the test set.

Support vector machines can be divided into three types: linear separable support vector machines, linear support vector machines, and nonlinear support vector machines. The algorithm flow can be summarized as follows: (1) input training data set; (2) select the kernel function; (3) build optimization equation based on kernel function; (4) solve the optimization equation to get the optimal separating hyperplane.

SVM parameters generally refer to the kernel function *K*, the slack variable *γ*, and the penalty parameter *C*, and the core parameter is the kernel function.

SVM relies on the kernel function to generate the best classification hyperplane in a high-dimensional space. The sample can be linearly separable in low-dimensional space to linearly separable in high-dimensional feature space using the kernel function, resulting in a linearly separable classifier training in high-dimensional space. Kernel techniques are used to learn nonlinear transformations in a high-dimensional space by implicitly using a kernel function. Currently commonly used kernel functions are [27] liner kernel, polynomial kernel, and radial basis kernel. The linear kernel function is most commonly employed in linear separability, with minimal parameters and quick moves. The Gaussian kernel function is another name for the radial basis kernel function. It is the most extensively utilized because it has high learning and generalization capabilities for any sample. The Gaussian kernel function will be used as the SVM model's kernel parameter in this research. There are two techniques for choosing the kernel function: one is to decide based on past information, and the other is to judge based on the cross-validation method's minimum error concept. If the sample's prior information is known ahead of time, the kernel function can be chosen directly based on that knowledge; RBF can typically be chosen directly as the kernel function if the prior knowledge is unknown.

The slack variable A is related to the selection of the kernel function *K*. In other words, if the kernel function is RBF, the slack variable *γ* will be considered. In SVM, the number of support vectors will increase as *γ* decreases. However, the time to train the model is directly proportional to the number of support vectors, which means that the more the support vectors are, the longer it takes to train the model. Therefore, the choice of slack variable *γ* is also very important.

The penalty parameter *C* represents the tolerance of the model to errors. A model with a large *C* value is prone to overfitting, and a model with a small *C* value is prone to underfitting. Therefore, the value of the penalty parameter *C* should not be too large or too small.

### 3.3. AdaBoost

Boosting algorithm is a set of integrated learning algorithms based on Probably Approximately Correct (PAC) learning theory [28]. The core idea is to build a robust classifier through several base classifiers. The base classifier, also called the weak classifier, refers to a classification model whose recognition accuracy is only slightly higher than random guessing; that is, the error rate is less than 50%. A robust classifier refers to a classification model with a high recognition accuracy rate and can be completed in a short time classification model. In 1996, Freund and Schapire proposed the famous AdaBoost [29] algorithm, which has become a typical boosting algorithm. In 2014, Chen Tianqi [30] proposed the XGBoost algorithm, which significantly improved the algorithm's efficiency and has been widely used in the industry. This article uses the former boosting algorithm. AdaBoost is also called an adaptive boosting algorithm, where the basic idea is to train several different classifiers based on the training set, here usually weak classifiers, and then integrate these classifiers to form a robust classifier, that is, the final classifier.

For a given training data set, where each sample point is composed of an instance *X* and a label *Y*, the algorithm steps of AdaBoost are as follows.

First, initialize the weight distribution of the training set as

(14) $$\begin{array}{c} \;D_{1}=\left(\;w_{11},\;w_{12},\ldots ,\;w_{1n}\right),\;w_{1i}=\frac{1}{n}. \end{array}$$

Here, it is assumed that each training sample in the data set has a uniform weight distribution, to ensure that the weak classifier can learn on the original data.

Second, for different values of *K*, repeat the following steps:

Learn on the training set with weight distribution  *D*_*k*_ to get a weak classifier:

(15) $$\begin{array}{c} \;G_{k}\left(x\right)=X⟶\left\{-1,\;+1\right\}. \end{array}$$

Calculate the recognition error rate of weak classifier  *G*_*k*_(*x*) on the training set:

(16) $$\begin{array}{c} e_{k}=P\left(G_{k}\left(x\right)\neq \;y_{i}\right). \end{array}$$

Calculate the coefficient of  *G*_*k*_(*x*):

(17) $$\begin{array}{c} \alpha_{k}=0.5*\text{ln}\left(\frac{1-e_{k}}{e_{k}}\right). \end{array}$$

Then, update the weight distribution. In the learning process, the AdaBoost algorithm will continuously update the weight distribution of the training samples, so that the samples play different roles in different weak classifiers.

Third, construct a linear combination of weak classifiers:

(18) $$\begin{array}{c} f\left(x\right)=\overset{K}{\underset{k=1}{\sum }}\alpha_{k}G_{k}\left(x\right). \end{array}$$

Synthesize the final strong classifier:

(19) $$\begin{array}{c} G\left(x\right)=\text{sign}\left(f\left(x\right)\right), \end{array}$$

where sign is defined as

(20) $$\begin{array}{c} \text{sign}\left(x\right)=\left\{\begin{array}{cc} +1, & x\geq 0\\ -1, & x<0 \end{array}\right.. \end{array}$$

The main advantages of the AdaBoost algorithm are that the model's classification accuracy is high and the model is not prone to overfitting. Various regression classification models can be employed as weak classifiers in the model learning process, which is quite flexible.

## 4. Experiments and Discussion

### 4.1. Data Sets

The data set of this experiment comes from a CT image library of a tertiary hospital, with a total of 10058 images, of which the number of positive samples (sick samples) is 5000, and the number of negative samples (normal samples) is 5058.

### 4.2. Evaluation Method and Indicators

To objectively evaluate the performance of the model, it is necessary to select an appropriate evaluation method. The cross-validation method is currently one of the most common model performance evaluation methods. The cross-validation method divides the data into two parts: a training set and a validation set. The training set is used to train the model, and the validation set is used to evaluate the model. The advantages of the cross-validation method are that it can prevent overfitting and underfitting and that the evaluation results obtained are convincing. The cross-validation method is mainly used for model parameter selection and performance evaluation of multiple models under the same data. Common cross-validation methods include K-fold cross-validation and leave-one-out cross-validation.

For classification models, the commonly used performance evaluation indicators are accuracy, precision rate, recall rate, and *F*_1_ score. The corresponding calculation formula is as follows:

(21) $$\begin{array}{c} \text{ACC}=\frac{\text{TP}+\text{TN}}{\text{TP}+\text{FP}+\text{FN}+\text{TN}},\\ \text{PRE}=\frac{\text{TP}}{\text{TP}+\text{FP}},\\ \text{REC}=\frac{\text{TP}}{\text{TP}+\text{FN}},\\ F_{1}=\frac{2*\text{PRE}*\text{REC}}{\text{PRE}+\text{REC}}. \end{array}$$

### 4.3. Logit-Based Diagnostic Model

The core of the Logit diagnosis model is the Logit regression model, which mainly uses Logit regression to predict whether the sample has a disease. Before constructing the Logit diagnostic model, the threshold of the Logit regression model needs to be determined. This paper uses the 5-fold cross-validation method to determine the threshold; that is, the data set is randomly divided into five parts. Then, the correct average rate of the 5 cross-validation models is calculated according to a given threshold. Finally, the maximum average correct rate is passed in principle, and the threshold *v* is selected. In this paper, the given threshold interval is [0.05, 0.1,…, 0.95], that is, an arithmetic sequence with an initial value of 0.05 and a step size of 0.05.

Through the 5-fold cross-validation method, the relationship between the average correct rate of the Logit diagnostic model and the threshold can be obtained as shown in Figure 1.

It can be found that when the threshold *v*=0.5, the average accuracy rate reaches the maximum value, which is close to 80%. Therefore, the threshold of the Logit regression model is set to 0.5. After determining the model's threshold, the correct rate, precision, recall, and score of the cross-validation model can be calculated using the 5-fold cross-validation method. Then, the correct average rate and the average score of the Logit diagnostic model can be calculated. The specific results are shown in Table 1.

The Logit regression diagnosis model has an average correct rate of 79.6% and an average *F*_1_ score of 47.5%. The diagnostic effect of the model is poor.

### 4.4. SVM-Based Diagnosis Model

The core of the SVM diagnosis model is the SVM classification model, which mainly uses SVM classification to predict whether the sample has a disease. Before constructing the SVM diagnosis model, three parameters of the SVM classification model need to be determined. Firstly, the kernel function needs to be determined. This paper chooses the most widely used Gaussian kernel function as the kernel function of the SVM classification model; then, the slack variables and penalty parameters are determined. In this paper, we use the 10-fold cross-validation method when determining the parameters.

First, according to the 10-fold cross-validation method, the optimal parameters can be obtained as *γ*=0.01, *C*=10. After the parameters of the model are determined, the accuracy, precision, recall, and *F*_1_ scores of the five cross-validation models can be calculated according to the 5-fold cross-validation method, and then the average accuracy rate and average *F*_1_ score of the SVM diagnostic model can be calculated in the middle. The specific results are shown in Table 2.

The SVM regression diagnosis model has an average correct rate of 89.0% and an average *F*_1_ score of 75.0%. The diagnostic effect of the model is good.

### 4.5. AdaBoost-Based Diagnosis Model

The core of the AdaBoost diagnostic model is the AdaBoost classification model, which mainly uses AdaBoost classification to predict whether the sample has a disease. Before constructing experiments with the AdaBoost diagnostic model, we first need to determine the number of weak classifiers *K* of the AdaBoost classification model. Generally, the number of classifiers *K* can be determined according to the convergence of the error rate of the classification model. The relationship between the error rate of the AdaBoost classification model and the number of classifiers is shown in Figure 2.

The error rate has begun to converge when the number of classifiers *K*=80. After determining the number of classifiers of the model, the correctness, precision, recall, and *F*_1_ scores of the five cross-validation models can be calculated according to the 5-fold cross-validation method, and then the average correctness and the average F1 score of the SVM diagnostic model can be calculated. Among them, the correct rate, precision rate, recall rate, and *F*_1_ score of the five cross-validation models are shown in Table 3.

The AdaBoost regression diagnosis model has an average correct rate of 90.0% and an average *F*_1_ score of 77.7%. The diagnostic effect of the model is excellent.

### 4.6. Comparison between Diagnostic Models

Based on the above analysis, the corresponding model is better than other models.

The average accuracy rate and average *F*_1_ score of the three diagnostic models are shown in Table 4.

The AdaBoost-based targeting model has the highest diagnostic accuracy and the best performance for rheumatic immune diseases as shown in Figure 3, Figure 4, and Figure 5.

## 5. Conclusions

This article focuses on the use of machine learning algorithms in the diagnosis of rheumatic immunological illnesses, as well as some practical implications for disease-assisted diagnosis and intelligent medical diagnosis. The following are the primary tasks achieved in this paper: We introduced the research foundation and relevance of disease-assisted diagnosis systems and intelligent medical diagnosis, as well as the current state of disease diagnosis research and machine learning development history. We introduced three popular machine learning algorithms: logistic regression, support vector machine classification, and adaptive boost classification, as well as the principles, procedures, benefits, and drawbacks of each model. We introduced the data sources and basic information for the case data, as well as the model performance evaluation methodologies and indicators. The rheumatic immune illness data set is used for the case data. The model parameters are chosen using the K-fold cross-validation approach, which is also used to evaluate the method. The accuracy, precision, recall, and model classification scores are among the evaluation metrics. The classification and diagnostic models are built using three algorithms: logistic regression, support vector machine classification, and adaptive boost classification. The diagnosis models are then evaluated based on the evaluation methodologies and indicators. The diagnostic model based on the AdaBoost algorithm has the best robustness, according to the evaluation results.

## Figures and Tables

**Figure 1:** The relationship between the average accuracy and the threshold.

**Figure 2:** The relationship between the error rate and the number of classifiers.

**Figure 3:** Comparison between different diagnostic models w.r.t. accuracy.

**Figure 4:** Comparison between different diagnostic models w.r.t. precision.

**Figure 5:** Comparison between different diagnostic models w.r.t. recall.

**Table 1:** Performance evaluation of the Logit diagnostic model.

Item	Acc (%)	Pre (%)	Rec (%)	*F*_1_ (%)
Pred1	78.3	66.8	34.9	45.8
Pred2	79.2	66.0	35.8	46.7
Pred3	80.3	70.8	36.8	48.0
Pred4	80.1	67.5	37.8	48.6
Pred5	80.0	66.9	38.5	48.6
Ave	79.6	67.6	36.8	47.5

**Table 2:** Performance evaluation of the SVM diagnostic model.

Item	Acc (%)	Pre (%)	Rec (%)	*F*_1_ (%)
Pred1	88.7	90.6	63.8	74.8
Pred2	88.8	89.1	62.7	73.6
Pred3	89.0	88.0	65.3	74.9
Pred4	89.1	89.7	66.9	76.8
Pred5	89.5	90.9	63.7	75.1
Ave	89.0	89.7	64.5	75.0

**Table 3:** Performance evaluation of the AdaBoost diagnostic model.

Item	Acc (%)	Pre (%)	Rec (%)	*F*_1_ (%)
Pred1	89.7	89.4	68.7	77.7
Pred2	89.2	85.9	67.9	75.9
Pred3	89.9	87.9	69.7	77.6
Pred4	90.6	89.3	70.5	78.9
Pred5	90.7	90.9	68.7	78.3
Ave	90.0	88.7	69.1	77.7

**Table 4:** Comparison between different diagnostic models.

Model	Logit (%)	SVM (%)	AdaBoost (%)
Acc	79.6	89.0	90.0
*F*_1_	47.5	75.0	77.7

## Data Availability

The data sets used and analyzed during the current study are available from the author upon reasonable request.
